The article "Virtual Simulation Design Facing Smart Payment Screen on the Background of Artificial Intelligence" was retracted in 2023. Reasons: signs of a paper mill; suspected computer-generated content; unreliable results or conclusions; concerns about the data.

# Virtual Simulation Design Facing Smart Payment Screen on the Background of Artificial Intelligence

**DOI:** 10.1155/2022/5336548

**Published:** 2022-10-08

**Authors:** Yan Li, Xiao Wang

**Affiliations:** Xi'an Fanyi University, Xi'an, Shaanxi 710105, China

## Abstract

In recent years, the rapid development of virtual simulation technology has become a hot topic among thousands of people. Virtual simulation has been used in education, transportation, anti-theft, and other fields, but it has not seen its application in the field of intelligent payment. This study designed an intelligent payment screen based on virtual simulation technology and evaluated the relevant performance. The evaluation results found that compared with the traditional payment screen, the use of smart payment screen for payment had the fastest improvement in security and the slowest improvement in usability, an increase of 4.2%; the youth group believed that the convenience of use of the smart payment screen based on virtual simulation technology has improved the fastest. The elderly group believed that the use of the smart payment screen based on virtual simulation technology had the slowest improvement in ease of use, an increase of 9.4%; the average payment time of each place has decreased, the average payment time of place 4 was the longest, and the average payment time of place 6 was the shortest, and it was concluded that the higher the payment success rate was, the shortest payment time was; in terms of the user's preference for the smart payment screen, it was concluded that 18:00 was the peak period for users to use the smart payment screen; in terms of risk assessment of using smart payment screens, it was concluded that compared with traditional payment screens, operational risk was reduced by 3.88%, credit risk was reduced by 4.67%, liquidity risk was reduced by 5.06%, and settlement risk was reduced by 6.01%. The design of the smart payment screen makes the user's payment more secure, and the payment risk is greatly reduced.

## 1. Introduction

The era of artificial intelligence has arrived, and artificial intelligence technology is used in speech recognition, autonomous driving, and smart cities in life. With the popularization of computer applications, artificial intelligence technology has also been applied and promoted. People are full of joy in the beautiful life brought by artificial intelligence, and at the same time they are eager to bring more convenience to life through artificial intelligence. In the field of payment, users also have new thinking about smart payment, people expect payment to be more secure, and hope to make new changes. In the recent years, mobile payment (MP) has become popular, and many different payment screens have emerged on the market. However, most of the current MPs have defects, such as poor security and weak system, and cannot meet people's daily payment needs. Moreover, in the environment of artificial intelligence, virtual simulation technology is also becoming mature and has been applied in various fields. In order to improve the security of smart payment and change the defects of current market payment, it is urgent to design a smart payment screen based on virtual simulation technology.

At this stage, the payment system and its technology are a hot topic, and many scholars have conducted research on intelligent payment. HHS Centers for Medicare & Medicaid Services described changes in the amounts and factors used to determine payment rates for Medicare services paid under the Medicare Hospital Outpatient Prospective Payment System and Medicare Ambulatory Surgery Center payment systems [1]. Layton et al. developed a measure of the efficiency consequences of price and benefit distortions under a particular payment system, building on previous research on the evaluation of health plan payment systems [2]. Feng et al. proposed a blockchain-based privacy-preserving payment mechanism, which enabled data sharing while ensuring the security of sensitive user information. This mechanism introduced a registration and data maintenance process based on blockchain technology, which realized the payment audit of privileged users while ensuring the anonymity of user payment data [3]. Mondal et al. introduced a generalized order-level inventory system that fully allowed late payments within various transaction credit intervals [4]. Barkhordari et al. conducted an experimental investigation of important factors influencing trust in Iran's electronic payment system. Research has found that both perceived security and trust have a positive impact on the use of electronic payment systems [5]. Tsao et al. explored the impact of dynamic discount-based credit payments on supply chain network design issues, also considered the time value of money, and applied cash flow discounting to formulate a model that determines the optimal replenishment cycle, selling price, and scope of influence for distribution centers while maximizing the present value of total profits [6]. Khalilzadeh et al. provided a comprehensive model to study the determinants of near field communication (NFC)-based MP technologies in the restaurant industry. The results showed that the proposed model provided about 20% more explanatory power and predictive accuracy than the original unified theoretical model of technology acceptance and use, and proved the impact of risk, safety, and trust on customers' intentions to use NFC-based MP technology in the restaurant environment [7]. To summarize, payment is an issue worthy of study, but there is currently no research on smart payment screens in the market.

Virtual simulation technology has played an indispensable role since the rapid development of information technology, and many scholars have conducted in-depth research on it. Cagnazzo used Sim&Size software to conduct virtual simulations to determine whether there would be an impact on technical, angiographic, and clinical outcomes after WEB treatment. It was found that virtual simulation with Sim&Size software appeared to be helpful in selecting an appropriate braided endo-bridge device for aneurysm treatment, thereby reducing intervention time, radiation dose, number of undeployed devices, and the need for corrective interventions [8]. Hudder et al. compared students studying neonatal assessment using virtual simulations with students in a traditional laboratory setting to assess students' knowledge, skills, satisfaction, self-confidence, and clinical judgment. Results showed that students' knowledge acquisition of neonatal assessment was greater when content and demonstrations were provided through virtual simulations, but student satisfaction and self-confidence were higher due to the opportunity to participate in live laboratory activities [9]. Mackenna et al. used an exploratory descriptive design for students to complete virtual simulations and then conducted self-reporting activities. The results showed that students demonstrated different levels of reflective thinking through self-reporting [10]. Mht et al. investigated whether the inclusion of virtual simulations in the required first-year self-care therapy course would affect the frequency of interactions, self-reported student confidence, and the performance of students reported by recipients during the second-year Introduction to Community Pharmacy Practice Experiences [11]. Fogg et al. used the clinical judgment scale to assess the effect of virtual simulations on students' self-perceived clinical judgment abilities. The results showed that virtual simulation was beneficial to students' learning and development of clinical judgment ability [12]. Padilha et al. assessed the ease and usefulness of clinical virtual simulations and the intention of emergency nurses to use clinical virtual simulations to improve their clinical reasoning skills for lifelong learning [13]. Verkuyl et al. delved into the advantages of self-reporting immediately after a virtual game simulation and the value of maximizing reflection by adding group debriefing [14]. Therefore, most of the researches were based on virtual simulation technology on medical treatment, education, and so on. It was rarely heard of its application in the field of smart payment. Based on this, this article adopted virtual simulation technology to simulate the design of intelligent payment screen.

In this article, the simulation technology was used to design an intelligent payment screen, and the security, usability, reliability, and convenience of the intelligent payment screen were compared with the traditional payment screen. At the same time, a survey of users' preference for the smart payment screen was conducted, and the possible risks of using the smart payment screen were evaluated in order to provide more possibilities for intelligent payment, enrich payment methods, and greatly improve the convenience of payment.

## 2. Algorithm of Virtual Simulation Technology

The first-order differential formula is set as:

(1) $$\begin{array}{c} \dot{Y}=F\left(t,Y\right). \end{array}$$

In the formula:

(2) $$\begin{array}{c} Y={\left(y_{1},y_{2},\cdots y_{n}\right)}^{T}, \end{array}$$

(3) $$\begin{array}{c} F={\left(f_{1}\left(t,Y\right),f_{2}\left(t,Y\right),\cdots f_{n}\left(t,Y\right)\right)}^{T}. \end{array}$$

(1) Fourth-order Runge–Kutta method.

*h* is a fixed step size, and the vector form of the fourth-order Runge–Kutta method at this time is:

(4) $$\begin{array}{c} Y_{n+1}=Y_{n}+\frac{h}{6}\left(K_{1}+2K_{2}+2K_{3}+K_{4}\right), \end{array}$$

(5) $$\begin{array}{c} K_{1}=F\left(t_{n},Y_{n}\right), \end{array}$$

(6) $$\begin{array}{c} K_{2}=F\left(t_{n}+\frac{h}{2},Y_{n}+\frac{h}{2}K_{1}\right), \end{array}$$

(7) $$\begin{array}{c} K_{3}=F\left(t_{n}+\frac{h}{2},Y_{n}+\frac{h}{2}K_{2}\right), \end{array}$$

(8) $$\begin{array}{c} K_{4}=F\left(t_{n}+\frac{h}{2},Y_{n}+\frac{h}{2}K3\right). \end{array}$$

The Taylor series expansion of *y*_*n*+1_ at *t*_*n*_ is performed:

(9) $$\begin{array}{c} y_{n+1}=y_{n}+\overset{r}{\underset{i=1}{\sum }}\frac{h^{i}}{i!}{y_{n}}^{\left(i\right)}+O\left(h^{r+1}\right). \end{array}$$

For $\dot{y}=\lambda y$, there is *y*^(*i*)^ = *λ*^*i*^*y*, and substitute it into the previous formula:

(10) $$\begin{array}{c} y_{n+1}=y_{n}\overset{r}{\underset{i=0}{\sum }}\frac{h^{i}}{i!}y_{n}^{\left(i\right)}+O\left(h^{r+1}\right). \end{array}$$

The stability condition of this formula is that the absolute value of the iteration coefficient is <1.

(11) $$\begin{array}{c} \left|\overset{r}{\underset{i=1}{\sum }}\frac{{\left(\lambda h\right)}^{i}}{i!}\right|<1. \end{array}$$

(2) Real-time Runge–Kutta formula.

(1) Real-time second-order Runge–Kutta method

(12) $$\begin{array}{c} Y_{n+1}=Y_{n}+{hK}_{2}, \end{array}$$

(13) $$\begin{array}{c} K_{1}=F\left(t_{n},Y_{n}\right), \end{array}$$

(14) $$\begin{array}{c} K_{2}=F\left(t_{n}+\frac{h}{2},Y_{n}+\frac{h}{2}K_{1}\right). \end{array}$$

(2) Real-time fourth-order Runge–Kutta method

(15) $$\begin{array}{c} Y_{n+1}=Y_{n}+\frac{h}{24}\left(-K_{1}+15K_{2}-5K_{3}+5K_{4}+10K_{5}\right), \end{array}$$

(16) $$\begin{array}{c} K_{1}=F\left(t_{n},Y_{n}\right), \end{array}$$

(17) $$\begin{array}{c} K_{2}=F\left(t_{n}+\frac{h}{5},Y_{n}+\frac{h}{5}K_{1}\right), \end{array}$$

(18) $$\begin{array}{c} K_{3}=F\left(t_{n}+\frac{2h}{5},Y_{n}+\frac{2h}{5}K_{1}\right), \end{array}$$

(19) $$\begin{array}{c} K_{4}=F\left(t_{n}+\frac{3h}{5},Y_{n}-\frac{2h}{5}K_{1}+{hK}_{2}\right), \end{array}$$

(20) $$\begin{array}{c} K_{5}=F\left(t_{n}+\frac{4h}{5},Y_{n}+\frac{3h}{10}K_{1}+\frac{h}{2}K_{4}\right). \end{array}$$

## 3. Virtual Simulation Design for Smart Payment Screen

### 3.1. Payment Tokenization

Payment tokenization technology is a security technology that is born to prevent information leakage. That is to say, it is a technical way to convert the sensitive information of financial institution users to form a corresponding token (Token), and use Token to replace the original sensitive information for information exchange during payment [15, 16]. This technology can effectively reduce the risk of sensitive information leakage, prevent financial losses, and protect the legitimate rights and interests of consumers. The smart payment screen designed in this article aims to use payment tokenization technology to ensure the payment security and convenience of those who use the smart payment screen. The bank card data and payment data stored in the terminal are encrypted and protected by the security module, and the user's identity is verified by biometric features to avoid payment data input. 3D modeling technology is used to build an immersive payment scene to design a standard payment solution that can not only improve the user experience but also ensure security to solve the industry's pain points. The specific design scheme is shown in Figure 1.

The payment tokenization system can effectively guarantee the payment security of those who use the smart payment screen, who show the token to the merchant, and then flow to the card issuer through different paths [17, 18]. The merchant's mark flows to two parties: one is to request the mark from the mark requester, this path flows to the mark management library, and finally flows to the card issuer due to the mark guarantee; on the other side, it flows through the token transfer to the acquirer, then to the card organization, and finally to the card issuer in the same way as the other path.

The payment tokenization system contains several important roles: (1) persons using smart payment screens: a smart payment screen will be held and the token can be streamed to the card issuer. (2) Card issuer: it owns the account relationship with the cardholder, owns the authorization, and ongoing risk management in the payment token ecosystem. (3) Merchant: it may be the recipient of the payment token in place of the PAN, or it may be the token requester. (4) Acquirer: all transactions will be handled in the same way as now, including authorization authentication, payment consumption, clearing, and exception handling.

### 3.2. Architecture Design of Smart Payment Screen

The design of smart payment screen needs to meet the security needs and practical needs of users, not only contracting institutions, card organizations, but also virtual reality (VR) equipment [19]. The specific architecture design of the smart payment screen is shown in Figure 2.

#### 3.2.1. Institution

Institution includes banking institutions and third-party institutions. Both are security carrier issuers, and their main functions are: controlling the master key of the primary security domain, assisting in the installation of “auxiliary security domains,” and managing the life cycle.

#### 3.2.2. Card Organization

The card organization includes three parts: trusted service, trust service provider (TSP), and online payment platform. Trusted services are interconnected with trusted service systems, such as operators and terminal manufacturers to provide banks with services, such as over-the-air card issuance and security module life cycle management; TSP provides payment tokenization services; online payment platforms provide online payment access, verify payment data, and accept transactions.

#### 3.2.3. VR Equipment

The security module is used to provide secure storage of financial information and secure access control, including the issuance and update of symmetric and asymmetric encryption algorithms and digital certificates, the dynamic issuance, deletion and update of bank financial data, the security isolation of financial data, and the provision of APIs for secure transactions. The security module includes four modules: access control, secure transmission, secure interface, and secure storage. The main component of the VR application part is the VR payment control. The VR payment control provides users with payment portals in VR scenarios, allowing users to select payment cards and discounts, use biometrics to authenticate user identities, dynamically generate ciphertext of payment data, and verify payment data and acceptance transactions through online payment platforms.

### 3.3. Security Module

The original intention of this article to design an intelligent payment screen based on the simulation technology is to improve the security of payment, so the security module is carefully designed. The security module includes access control, key exchange, secure interface, and secure communication [20]. The specific architecture diagram is shown in Figure 3.

#### 3.3.1. Access Control

Access control restricts the access of the access subject to the object, thus ensuring the effective use and management of data resources within the legal scope. This design effectively protects the rights and interests of the visiting subject, protects its legal status from being infringed, and also protects the user's payment security. For unknown and illegal software and hardware resources, it is impossible to intrude into the payment system of the visiting subject without any reason, and the user's access security is greatly guaranteed.

#### 3.3.2. Key Exchange

Simply put, key exchange is to use an asymmetric encryption algorithm to encrypt a symmetric key to ensure the security of transmission, and then use a symmetric key to encrypt data. The key exchange guarantees the user's payment security to a large extent. The user's payment data can be encrypted to a large extent through this method, thus preventing the attack of unscrupulous data thieves.

#### 3.3.3. Security Interface

The security interface ensures the security of user data, and prevents malicious calls to the interface by third parties and requests from being modified during transmission. The design of the security interface makes users feel more secure in payment and the use of the smart payment screen.

#### 3.3.4. Secure Communication

Secure communication guarantees the security of the channel between the communication endpoints, with both confidentiality and integrity. Confidentiality is guaranteed with encryption, and integrity is guaranteed with message authentication codes. This not only ensures that user data is private and confidential, and will not be viewed by listeners using network monitoring software, but also protects user data from unauthorized or malicious modification during transmission. The setting of secure communication greatly protects the user's payment security.

## 4. Virtual Simulation Design Experiment for Smart Payment Screen

This article design an intelligent payment screen based on virtual simulation technology and puts it into use. The safety, usability, and reliability of the payment using the smart payment screen and the payment using the traditional payment screen were compared by using the VR payment scene in order to test whether the payment using the smart payment screen can achieve the effect of people's expected payment, and whether it can meet the needs of large-scale use in the market. The test results are recorded in Table 1 and Figure 4.

According to Table 1 and Figure 4, it can be seen that the payment security, usability, and reliability of using the smart payment screen are improved compared to the payment using the traditional payment screen. Security has increased by 19.2%, which is the fastest improvement, reliability has increased by 11.1%, and availability has increased by 4.2%, which is the slowest improvement. It can be seen that the use of the smart payment screen based on virtual simulation technology can greatly improve the security of payment, but the usability of the smart payment screen needs to be further improved to meet the needs of more consumers.

The most important purpose of the design of the smart payment screen is to improve the convenience of payment, make the payment method more convenient for people's life, and let the life get a better consumption experience due to smart payment. Therefore, this study selected different stages of the population and selected representatives to test the convenience of the smart payment, and compared it with the traditional payment. The test results are shown in Figure 5.

It can be seen from Figure 5 that in the survey on the convenience of use of the smart payment screen based on virtual simulation technology, teenagers and young people believe that the convenience of use of the smart payment screen based on virtual simulation technology is improved rapidly. The youth group believes that the convenience of use of the smart payment screen based on virtual simulation technology has improved the fastest, with an increase of 22.8%; the middle-aged and elderly groups believe that the convenience of use of the smart payment screen based on virtual simulation technology has been improved slowly, and they believe that the convenience of use of the smart payment screen based on virtual simulation technology has improved the fastest. The elderly group believes that the use of the smart payment screen based on virtual simulation technology has the slowest improvement in ease of use, an increase of 9.4%. The reason is that the majority of young people have a strong ability to accept new things, and they do not feel burdened by the use of the intelligent payment screen based on virtual simulation technology, but only feel novel; however, for the elderly, smart payment methods are a burden, and they cannot use smart payment screens well.

Payment convenience is a concept proposed that is relative to traditional paper currency payment. Compared with paper currency payment, MP only needs to carry a mobile phone instead of holding a lot of banknotes, thus enhancing the convenience of payment. There are two important indicators for evaluating the convenience of payment: first is the time cost of the payment process. The shorter the payment time is, the better the convenience of payment is; another important evaluation indicator related to the convenience of payment is the payment success rate. Due to the complexity of payment methods, many users may have low payment success rates due to improper operation or unfamiliarity with payment software, which greatly reduces payment efficiency and violates the original intention of payment convenience. Therefore, it is necessary to test the payment success rate to improve the convenience and efficiency of payment. Based on this, in order to investigate the convenience of using the smart payment screen based on virtual simulation technology, this study conducted an experimental investigation on two factors that affected its convenience. This experiment randomly selected 6 places that used the intelligent payment screen based on virtual simulation technology, and conducted a follow-up investigation on them, and compared it with the traditional MP screen. The test results are shown in Figures 6 and 7.

It can be seen from Figure 6 that the average payment duration of using the smart payment screen based on virtual simulation technology in various places is reduced compared to the average payment duration of using the traditional payment screen. The overall trend is roughly the same. Location 4 has the longest average payment time and location 6 has the shortest average payment time. It can be seen that the fundamental reason for the difference in the average payment time of each place is the difference in the flow of people and the network system of each place. Correspondingly, the reason can be found from Figure 7. The higher the payment success rate is, the shorter the payment time is.

In order to understand the user's preference for the smart payment screen, this article investigated the frequency of users using the smart payment screen. Location 4 was selected as the subjects of this experiment. Since the opening time of place 4 is from 10:00 to 20:00, five points were selected for this survey during this time period, and the survey results of users using the smart payment screen at different time points were recorded in Figure 8.

It can be seen from Figure 8 that 18:00 is the peak period for users to use the smart payment screen. Most people tend to use the smart payment screen at this point in time. Therefore, it is necessary to make preparations for the payment environment at this point in time, to ensure the smoothness of the network and the system to keep running well, to prevent the system from crashing and bring a bad payment experience to users.

The use of smart payment screens makes payment safe and convenient, but it cannot be denied that the use of smart payment screens also has certain risks. There may be operational risks in the use of smart payment screens, such as electronic pickpockets, online fraud, online hacking, credit risks, liquidity risks, and settlement risks. In order to avoid risks in the payment process and to improve the security of payment, this experiment evaluated the possible risks in the use of smart payment screens and compared them with traditional payment screens. *A* represents using the traditional payment screen, *B* represents using the smart payment screen, and the evaluation results are shown in Figure 9.

It can be seen from Figure 9 that the use risk of the smart payment screen is greatly reduced compared to the use risk of the traditional payment screen. Operational risk was reduced by 3.88%, credit risk by 4.67%, liquidity risk by 5.06%, and settlement risk by 6.01%. Users no longer have to worry about the risks of using smart payment screens, and merchants no longer have to provide users with unnecessary operations to reduce user experience, thereby improving corporate competitiveness.

## 5. Advantages and Disadvantages of Virtual Simulation Design for Smart Payment Screen

### 5.1. Advantages of Virtual Simulation Design for Smart Payment Screens

#### 5.1.1. Payment Is More Convenient

The use of this smart payment screen makes the payment more convenient and the payment coverage is wide. Users' experience is stronger. Due to the use of smart payment screens, it is supported by virtual simulation technology. In terms of information auditing security, accurate identification can be achieved and the error rate can be reduced. It can almost be said to eliminate any impostor speculators and greatly improve the accuracy of information comparison. Moreover, the improvement of the algorithm will allow the payment process to be completed in a very short time, and the user experience will be better. Compared with traditional payment screens, they are more likely to accept this efficient and convenient payment screen.

#### 5.1.2. Payment Risk Is Reduced

The use of virtual simulation technology brings security to payment, and users are more willing to use the smart payment screen to pay. Compared with using a traditional payment screen, the use of the smart payment screen greatly reduces the payment risk. Consumers can complete the payment at any time and anywhere; the user only needs to connect the mobile phone or tablet with the smart payment terminal to complete the payment operation, which solves the problem of user privacy leakage during the payment process, thereby greatly improving the payment security.

### 5.2. Disadvantages of Virtual Simulation Design for Smart Payment Screens

The design of the smart payment screen still has some shortcomings, and it is a burden for the elderly users to use the smart payment screen. Therefore, the design of the smart payment screen needs to increase the use module for the elderly, so that this part of the group can also feel the convenience of using the smart payment screen and enhance their user experience.

## 6. Conclusions

In the context of artificial intelligence, this study designed an intelligent payment screen based on virtual simulation technology, compared it with the traditional payment screen, and evaluated the relevant content. In the performance test of the use of smart payment screens and traditional payment screens, it was concluded that the payment security, usability, and reliability of using smart payment screens were improved compared with those of traditional payment screens. The security has been improved by 19.2%, which was the fastest improvement, the reliability has been improved by 11.1%, and the availability has been improved by 4.2%, which was the slowest improvement; in the survey on the convenience of use of the smart payment screen based on virtual simulation technology, the youth group believed that the convenience of use of the smart payment screen based on virtual simulation technology has improved the fastest, with an increase of 22.8%. The elderly group believed that the use of the smart payment screen based on virtual simulation technology had the slowest improvement in ease of use, an increase of 9.4%; in terms of the payment duration of the use of the intelligent payment screen based on the virtual simulation technology, the average payment duration of each place was reduced. The average payment time of place 4 was the longest, and the average payment time of place 6 was the shortest, and it was concluded that the higher the payment success rate was, the shortest payment time was; in terms of the user's preference for the smart payment screen, it was concluded that 18:00 was the peak period for users to use the smart payment screen; in terms of risk assessment of using smart payment screens, it was concluded that compared with traditional payment screens, operational risk was reduced by 3.88%, credit risk was reduced by 4.67%, liquidity risk was reduced by 5.06%, and settlement risk was reduced by 6.01%.

## Figures and Tables

**Figure 1:** Payment markup structure.

**Figure 2:** Technical architecture diagram.

**Figure 3:** Security policy system.

**Figure 4:** Comparison of two different payment methods.

**Figure 5:** Convenience comparison of two different payment methods.

**Figure 6:** Average duration of two payment methods.

**Figure 7:** Payment success rate of two payment methods.

**Figure 8:** The number of times users use the smart payment screen in different time periods.

**Figure 9:** Risk assessment for use of different payment screens.

**Table 1:** Comparison of the advantages of smart payment and traditional payment.

	Traditional payment	Smart payment
Safety (%)	59.4	68.6
Availability (%)	61.7	65.9
Reliability (%)	68.4	79.5

## Data Availability

Data supporting this research article are available from the corresponding author or first author on reasonable request.

## References

[1] HHS Centers for Medicare & Medicaid Services (CMS) (2017). Medicare program: hospital outpatient prospective payment and ambulatory surgical center payment systems and quality reporting programs. Final rule with comment period. *Federal Register*.

[2] Layton T. J., Ellis R. P., Mcguire T. G. l. (2017). Measuring efficiency of health plan payment systems in managed competition health insurance markets. *Journal of Health Economics*.

[3] Feng G., Zhu L., Meng S. (2018). A blockchain-based privacy-preserving payment mechanism for vehicle-to-grid Networks. *IEEE Network*.

[4] Mondal B., Garai A., Roy T. K. (2021). Optimization of generalized order-level inventory system under fully permissible delay in payment. *RAIRO—Operations Research*.

[5] Barkhordari M., Nourollah Z., Mashayekhi H., Mashayekhi Y., Ahangar M. S. (2017). Factors influencing adoption of e-payment systems: an empirical study on Iranian customers. *Information Systems and e-Business Management*.

[6] Tsao Y. C., Setiawati M., Vu T. L. (2021). Designing a supply chain network under a dynamic discounting-based credit payment program. *RAIRO—Operations Research*.

[7] Khalilzadeh J., Ozturk A. B., Bilgihan A. (2017). Security-related factors in extended UTAUT model for NFC based mobile payment in the restaurant industry. *Computers in Human Behavior*.

[8] Cagnazzo F. (2022). Comparison of woven endobridge device sizing with conventional measurements and virtual simulation using the sim & size software: a multicenter experience. *Journal of Neuroradiology*.

[9] Hudder K., Buck-Mcfadyen E., Regts M. (2021). A quasi-experimental study comparing virtual simulation to lab-based learning of newborn assessment among nursing students. *Clinical Simulation in Nursing*.

[10] Mackenna V., Díaz D. A., Chase S. K. (2021). Self-debriefing after virtual simulation: measuring depth of reflection. *Clinical Simulation in Nursing*.

[11] Mht A., Nr A., Kck A. (2020). Impact of virtual simulation in self-care therapeutics course on introductory pharmacy practice experience self-care encounters. *Currents in Pharmacy Teaching and Learning*.

[12] Fogg N., Kubin L., Wilson C. E., Trinka M. (2020). Using virtual simulation to develop clinical judgment in undergraduate nursing students. *Clinical Simulation in Nursing*.

[13] Padilha J. M., Ribeiro A., Rosa J., Marques D., Machado P. P. (2020). Clinical virtual simulation as lifelong learning strategy—Nurse’s verdict. *Clinical Simulation in Nursing*.

[14] Verkuyl M., Lapum J. L., St-Amant O., Hughes M., Romaniuk D., McCulloch T. (2020). Exploring debriefing combinations after a virtual simulation. *Clinical Simulation in Nursing*.

[15] Zhang J., Luximon Y. (2021). A quantitative diary study of perceptions of security in mobile payment transactions. *Behaviour & Information Technology*.

[16] You J., Han M., Kim K. (2018). A study on method for bypassing verification function by manipulating return value of android payment application’s security solution. *Journal of the Korea Institute of Information Security and Cryptology*.

[17] Nouri A., Hosseini S. H. (2017). Payment minimisation auction with security constraints. *IET Generation Transmission & Distribution*.

[18] Tomkies M. C., Valentine L. P. (2018). Virtual currency: a commodity, property, security, or payment substitute. *Banking & Financial Services Policy Report*.

[19] Hu L. (2019). E-commerce trade consumption payment security and privacy based on improved B2C model. *International Journal of Network Security*.

[20] Wan S., Yang G., Qi L., Li L., Yan X., Lu Y. (2019). Multiple security anti-counterfeit applications to QR code payment based on visual secret sharing and QR code. *Mathematical Biosciences and Engineering*.

